The article "Investigation on Psychological Status and Job Burnout of Managers in Petroleum Enterprises" was retracted in 2023. Reasons: suspected computer-generated content; unreliable results or conclusions; concerns about the data; concerns about the results or conclusions.

# Investigation on Psychological Status and Job Burnout of Managers in Petroleum Enterprises

**DOI:** 10.1155/2022/4798220

**Published:** 2022-02-09

**Authors:** Bin Liu, Jijun Zhang

**Affiliations:** ^1^School of Economics and Management Southwest Petroleum University, Chengdu, China; ^2^School of Administration, Chengdu University of Traditional Chinese Medicine, Chengdu, China

## Abstract

Primarily in this paper, we have thoroughly investigated the psychological status and job burnout of managers in petroleum enterprises. For this purpose, we have assumed managers in petroleum enterprises as the research objects, whereas the overall sampling method was adopted from January 2019 to June 2020. A total of 240 questionnaires were sent out and 236 valid questionnaires were received with a recovery rate of 98.33%. The research objects' general information, psychological health status, and job burnout level were investigated. Among the 236 management personnel in petroleum enterprises, 212 (89.83%) were male and 24 (10.17%) were female. The average age was (40.28 ± 7.07) years old, and the number of people aged 40–49 was the largest, accounting for 52.12%; 84.32% were in marriage; regular college or above accounted for 81.78%; no smoking or occasional smoking in the last one year was 52.97%; not drinking in the last year was 34.75%; and 60.17% of managers in petroleum enterprises never or occasionally exercise. 121 (51.27%) suffered from high burnout due to emotional exhaustion, 125 (52.97%) suffered from high burnout due to emotional alienation, and 139 (58.90%) suffered from high burnout due to reduced sense of achievement. The scores of somatization, obsessive symptoms, depression, anxiety, and terror of the respondents were significantly higher than the normal levels of domestic adults. The differences were statistically significant (*P* < 0.05); there was no statistical significance in the scores of the other four factors compared with the national norm (*P* > 0.05). The phenomenon of job burnout and some psychological health problems existed in the managers in petroleum enterprises. The incidence of psychological evaluation was higher than that of the national norm, and the level of psychological health could predict the job burnout of petroleum enterprise managers.

## 1. Introduction

In recent years, some petroleum enterprises have experienced a lot of loss of management personnel and low work efficiency, the main reason is that the income of managers is very uncertain and there are more and more opportunities for excellent managers to flow [1, 2]. Previous studies have shown that there are many high risk factors of job burnout and more and more serious psychological health problems among managers of petroleum enterprises [3]. Under high pressure, managers in petroleum enterprises are prone to psychological problems, if not adjusted in time, it is easy to cause fatigue, emotional alienation, poor nursing quality, and other job burnout [4]. Especially under the background of the system reform of petroleum enterprises, the job burnout of managers personnel in petroleum enterprises is more common, and its severity is worrying [5, 6]. The job burnout state of managers in petroleum enterprises will affect their own health and development, which may increase the risk of sleep disorders, hypertension, myocardial infarction, and even suicide; it will also cause serious negative social impacts such as the loss of management personnel of petroleum companies and resignation [7]. The current situation of occupational burnout and mental health of managers in petroleum enterprises, the influence of factors, and the relationship between them are all worth exploring and researching [8]. However, there are few studies on the job burnout and psychological health of this population, and limited studies have shown that the job burnout and psychological health problems of managers in petroleum enterprises are more serious [9, 10]. This study focuses on how to reduce the occurrence of burnout of managers in petroleum enterprises as a foothold to carry out related research.

In this paper, we have thoroughly investigated the psychological status and job burnout of managers in petroleum enterprises. For this purpose, we have assumed managers in petroleum enterprises as the research objects, whereas the overall sampling method was adopted from January 2019 to June 2020. A total of 240 questionnaires were sent out and 236 valid questionnaires were received with a recovery rate of 98.33%. The research objects' general information, psychological health status, and job burnout level were investigated. Among the 236 management personnel in petroleum enterprises, 212 (89.83%) were male and 24 (10.17%) were female. The average age was (40.28 ± 7.07) years old, and the number of people aged 40–49 was the largest, accounting for 52.12%; 84.32% were in marriage; Regular college or above accounted for 81.78%; no smoking or occasional smoking in the last one year was 52.97%; not drinking in the last year was 34.75%; and 60.17% of managers in petroleum enterprises never or occasionally exercise. 121 (51.27%) suffered from high burnout due to emotional exhaustion, 125 (52.97%) suffered from high burnout due to emotional alienation, and 139 (58.90%) suffered from high burnout due to reduced sense of achievement. The scores of somatization, obsessive symptoms, depression, anxiety, and terror of the respondents were significantly higher than the normal levels of domestic adults. The differences were statistically significant (*P* < 0.05); there was no statistical significance in the scores of the other four factors compared with the national norm (*P* > 0.05).

The remaining sections or portions of this paper are organized as follows.

In subsequent section, the proposed methods implementation plan is described in detail along with definition of the various supportive parameters. Experimental and simulation results, both on the generated and benchmark data, were performed and presented a comparative study. A detailed discussion section is provided which is followed by the summary of the whole manuscript in the form of conclusion. Finally, references which are cited in the paper are presented.

## 2. Proposed Mechanism: Materials and Methods

### 2.1. General Information

With managers in petroleum enterprises as the research objects, the research was carried out with the approval of the ethics committee of our unit.

Inclusion criteria:

1. Petroleum enterprise management
2. Signed informed consent

Exclusion criteria:

1. Unwilling to participate in the survey
2. The working time was less than 1 year

### 2.2. Methodology: Implementation Plan

From January 2019 to June 2020, the overall sampling method was adopted. A total of 240 questionnaires were distributed and 236 valid questionnaires were returned, with a recovery rate of 98.33%.

### 2.3. Observational Index

The research objects' general information, psychological health status, and job burnout level were investigated.

1. General information: self-made individual characteristics questionnaire was used to collect the general information of the subjects, including gender, age, marital status, educational background, smoking status, alcohol consumption status, and exercise status.
2. Job burnout level: using the Maslach Job Burnout Scale [11]. The scale includes three dimensions: emotional alienation, emotional exhaustion, and reduced sense of achievement. There were 22 items, each of which was scored on a seven-point scale. Low burnout included emotional exhaustion score less than 19 points, emotional alienation score less than 6 points, and reduced sense of achievement score more than 34 points; moderate burnout included emotional exhaustion scores ranging from 19 to 26, emotional alienation scores ranging from 6 to 9, and a reduced sense of accomplishment of 26 to 34; high burnout included emotional exhaustion scores greater than 26, emotional alienation scores greater than 9, and reduced sense of accomplishment scores less than 26.
3. Psychological health status: SCL-90 Self-Rating Scale [12] included somatization (12 items), interpersonal sensitivity (9 items), depression (13 items), obsessive symptoms (10 items), anxiety (10 items), hostility (6 items), paranoia (6 items), terror (7 items), and psychosis (10 items); the other seven items reflect participants' sleep and diet. Each item was scored on a 5-point scale, with a total score of over 160 points, a single factor score ≥2 indicated that the tester had symptoms related to the factor, and the number of items with a score ≥2 indicated the number of positive items with symptoms.

### 2.4. Statistical Method

The analysis was performed using SPSS 19.0 software package. Measurement data were expressed as (*x* ± *s*), and *P* < 0.05 indicated statistically significant difference.

## 3. Results and Evaluations

### 3.1. Result of General Information

Among the 236 management personnel in petroleum enterprises, 212 (89.83%) were male and 24 (10.17%) were female. The average age was (40.28 ± 7.07) years old, and the number of people aged 40–49 was the largest, accounting for 52.12%; 84.32% were in marriage; regular college or above accounted for 81.78%; no smoking or occasional smoking in the last one year was 52.97%; not drinking in the last year was 34.75%; and 60.17% of managers in petroleum enterprises never or occasionally exercise. Result of general information is shown in Table 1.

### 3.2. Result of Job Burnout Level

121(51.27%) suffered from high burnout due to emotional exhaustion, 125 (52.97%) suffered from high burnout due to emotional alienation, and 139 (58.90%) suffered from high burnout due to reduced sense of achievement. Result of job burnout is shown in Table 2.

### 3.3. Result of Psychological Health Status

The scores of somatization, obsessive symptoms, depression, anxiety, and terror of the respondents were significantly higher than the normal levels of domestic adults. The differences were statistically significant (*P* < 0.05). There was no statistical significance in the scores of the other four factors compared with the national norm (*P* > 0.05). Result of psychological health status is shown in Table 3.

## 4. Discussion

The concept of job burnout was first put forward by the famous American psychologists Jackson and Maslach in 1984 [13]. In 2001, Maslach summarized that “job burnout” refers to a kind of comprehensive syndrome characterized by excessive physical and mental consumption and energy exhaustion under long-term work pressure [14]. Studies have shown that there is a high proportion of job burnout and energy exhaustion among managers of petroleum enterprises, which has a negative impact on ensuring the management quality of petroleum enterprises and the personal career development of managers to varying degrees [15, 16]. The level of emotional exhaustion, emotional alienation, and reduced sense of accomplishment of managers in petroleum enterprises is poor, indicating that managers in petroleum enterprises consume a lot of physical and psychological functions in corporate management work, aggravating their own sense of exhaustion, and reducing their sense of accomplishment causes oil company managers to show symptoms such as indifference, hostility, and lack of compassion [17]. Emotional exhaustion and high burnout suggest that the managers of petroleum enterprises have a deep sense of identity for the excessive consumption of their emotional and physiological functions; emotional alienation and high burnout indicate the objective response of managers of petroleum enterprises in enterprise management [18]; the reduced sense of achievement and high burnout indicate that the managers of petroleum enterprises no longer have enthusiasm for their work, their self-perception ability decreases, and they are more inclined to take care of their own negative critics [19, 20]. Existing research results reflect the current situation of psychological health and job burnout of managers in petroleum enterprises to a certain extent, revealing that job burnout is significantly positively correlated with mental health status, and mental health level can be used to predict the occurrence of job burnout [21]. Therefore, it is necessary to pay more attention to the managers in petroleum enterprises, enhance their career sense of achievement, and balance the relationship between life and work of the managers in petroleum enterprises, pay attention to the physical and mental health of managers in petroleum enterprises, create a harmonious working atmosphere between managers and ordinary employees in petroleum enterprises, and reduce the job burnout of managers in petroleum enterprises [22, 23]. The job burnout of the managers in petroleum enterprises will also bring a lot of negative effects to the society [24].

This study showed that

1. Among the 236 management personnel in petroleum enterprises, 212 (89.83%) were male and 24 (10.17%) were female. The average age was (40.28 ± 7.07) years old, and the number of people aged 40–49 was the largest, accounting for 52.12%; 84.32% were in marriage; regular college or above accounted for 81.78%; no smoking or occasional smoking in the last one year was 52.97%; not drinking in the last year was 34.75%; and 60.17% of managers in petroleum enterprises never or occasionally exercise.
2. 121 (51.27%) suffered from high burnout due to emotional exhaustion, 125 (52.97%) suffered from high burnout due to emotional alienation, and 139 (58.90%) suffered from high burnout due to reduced sense of achievement.
3. The scores of somatization, obsessive symptoms, depression, anxiety, and terror of the respondents were significantly higher than the normal levels of domestic adults. The differences were statistically significant (*P* < 0.05); there was no statistical significance in the scores of the other four factors compared with the national norm (*P* > 0.05).

## 5. Conclusion

Primarily in this paper, we have thoroughly investigated the psychological status and job burnout of managers in petroleum enterprises. For this purpose, we have assumed managers in petroleum enterprises as the research objects, whereas the overall sampling method was adopted from January 2019 to June 2020. A total of 240 questionnaires were sent out and 236 valid questionnaires were received with a recovery rate of 98.33%. The research objects' general information, psychological health status, and job burnout level were investigated. Among the 236 management personnel in petroleum enterprises, 212 (89.83%) were male and 24 (10.17%) were female. The average age was (40.28 ± 7.07) years old, and the number of people aged 40–49 was the largest, accounting for 52.12%; 84.32% were in marriage; regular college or above accounted for 81.78%; no smoking or occasional smoking in the last one year was 52.97%; not drinking in the last year was 34.75%; and 60.17% of managers in petroleum enterprises never or occasionally exercise. 121 (51.27%) suffered from high burnout due to emotional exhaustion, 125 (52.97%) suffered from high burnout due to emotional alienation, and 139 (58.90%) suffered from high burnout due to reduced sense of achievement. The scores of somatization, obsessive symptoms, depression, anxiety, and terror of the respondents were significantly higher than the normal levels of domestic adults. The differences were statistically significant (*P* < 0.05); there was no statistical significance in the scores of the other four factors compared with the national norm (*P* > 0.05). In conclusion, the phenomenon of job burnout and some psychological health problems existed in the managers in petroleum enterprises. The incidence of psychological evaluation was higher than that of the national norm, and the level of psychological health could predict the job burnout of petroleum enterprise managers.

## Figures and Tables

**Table 1:** Result of general information.

Projects		Number	Rate (%)
*Gender*	Male	212	89.83
	Female	24	10.17

*Age*	<30	20	8.47
	30–39	62	26.27
	40–49	123	52.12
	≥50	31	13.14

*Marital status*	In the marriage	199	84.32
	Not in marriage	37	15.68

*Educational background*	Senior high school and below	3	1.27
	Junior college	40	16.95
	Regular college course	152	64.41
	Master degree or above	41	17.37

*Smoking status*	No smoking or occasional smoking in the last one year	125	52.97
	Smoking frequently in the past year	111	47.03

*Alcohol consumption status*	Not drinking in the last year	82	34.75
	Drinking frequently in the past year	154	62.25

*Exercise status*	Never exercise or exercise occasionally	142	60.17
	Exercise regularly	94	39.83

**Table 2:** Result of job burnout.

Project	Number	Emotional alienation	Emotional exhaustion	Reduced sense of achievement
Low burnout	236	36(15.25)	37(15.68)	32(13.56)
Moderate burnout	236	75(31.78)	78(33.05)	65(27.54)
High burnout	236	125(52.97)	121(51.27)	139(58.90)

**Table 3:** Result of psychological health status.

Factors	Respondents	National norm	*t*	*P*
Somatization	1.37 ± 0.48	1.26 ± 0.35	2.314	<0.05
Interpersonal sensitivity	1.56 ± 0.49	1.54 ± 0.52	0.326	>0.05
Depression	1.54 ± 0.59	1.45 ± 0.48	2.526	<0.05
Obsessive symptoms	1.67 ± 0.57	1.53 ± 0.49	2.781	<0.05
Anxiety	1.38 ± 0.51	1.24 ± 0.35	2.284	<0.05
Hostility	1.43 ± 0.36	1.18 ± 0.31	1.446	>0.05
Paranoia	1.34 ± 0.52	1.32 ± 0.46	0.346	>0.05
Terror	1.21 ± 0.45	1.12 ± 0.32	2.072	<0.05
Psychosis	1.24 ± 0.33	1.18 ± 0.31	1.467	>0.05

## Data Availability

The data used to support the findings of this study are included within the article.
